# High-Frequency Vibrating Stimuli Using the Low-Cost Coin-Type Motors for SSSEP-Based BCI

**DOI:** 10.1155/2022/4100381

**Published:** 2022-08-25

**Authors:** Keun-Tae Kim, Junhyuk Choi, Ji Hyeok Jeong, Hyungmin Kim, Song Joo Lee

**Affiliations:** ^1^Bionics Research Center, Biomedical Research Division, Korea Institute of Science and Technology, Seoul 02792, Republic of Korea; ^2^Department of Brain and Cognitive Engineering, Korea University, Seoul 02841, Republic of Korea; ^3^Division of Bio-Medical Science & Technology, KIST School, Korea University of Science and Technology, Seoul 02792, Republic of Korea

## Abstract

Steady-state somatosensory-evoked potential- (SSSEP-) based brain-computer interfaces (BCIs) have been applied for assisting people with physical disabilities since it does not require gaze fixation or long-time training. Despite the advancement of various noninvasive electroencephalogram- (EEG-) based BCI paradigms, researches on SSSEP with the various frequency range and related classification algorithms are relatively unsettled. In this study, we investigated the feasibility of classifying the SSSEP within high-frequency vibration stimuli induced by a versatile coin-type eccentric rotating mass (ERM) motor. Seven healthy subjects performed selective attention (SA) tasks with vibration stimuli attached to the left and right index fingers. Three EEG feature extraction methods, followed by a support vector machine (SVM) classifier, have been tested: common spatial pattern (CSP), filter-bank CSP (FBCSP), and mutual information-based best individual feature (MIBIF) selection after the FBCSP. Consequently, the FBCSP showed the highest performance at 71.5 ± 2.5% for classifying the left and right-hand SA tasks than the other two methods (i.e., CSP and FBCSP-MIBIF). Based on our findings and approach, the high-frequency vibration stimuli using low-cost coin motors with the FBCSP-based feature selection can be potentially applied to developing practical SSSEP-based BCI systems.

## 1. Introduction

In recent few decades, noninvasive brain-computer interfaces (BCIs) have been applied for assisting the real-life of people with paralysis, such as spinal cord injury or amyotrophic lateral sclerosis [1, 2]. Electroencephalogram- (EEG-) based BCIs have been employed to control external devices such as lower-limb exoskeletons [3, 4], robotic arms [5], and spellers [6, 7]. Various exogenous (e.g., P300 [8] and steady-state visual evoked potential (SSVEP) [9]) and endogenous (e.g., motor imagery (MI) [10]) EEG paradigms were widely used for recognizing the user's intentions. However, the aforementioned paradigms have some limitations. For example, P300 and SSVEP interfaces require visual attention to the flickering stimulation, and the intensive training session is essential to the MI protocol. As various BCI applications have been expanded to activities of daily living (ADLs) [11], BCI operators are required to be aware of the outer surroundings instead of laying down or sitting still to engage one's whole attention to the interfaces. According to the recent review studies, most of the developed BCI-based communication devices still rely on the user's visual attention [11, 12]. Since 70% of human sensory receptors are related to vision [13], the visually induced BCI paradigms could distract or at least cause fatigue to the subjects.

Recently, a steady-state somatosensory evoked potential (SSSEP) via selective attention (SA) task has been alternatively studied to take advantage of both exogenous and endogenous BCI paradigms [14–17]. The SSSEP is a brain response eliciting evoked potentials at the same frequency as the tactile stimulation given at a specific frequency [15]. The SSSEP-BCI has the advantage of reducing visual load and interfacing with extra devices conveniently. The SSSEP was applied to BCI for the first time in 2006 [17]. Müller-Putz et al. reported that SA to a specific stimulus could modulate the induced SSSEP and exploited this potential to implement the BCI. However, in previous studies, SSSEP has been studied only with a focus on the low-frequency range (<41 Hz) [14–17].

Considering real-life appliances such as smartphones that usually use high-frequency vibration, investigating high-frequency SSSEP-based BCI could potentially have a greater impact on controlling real-life appliances using BCI. In addition to expanding the application of SSSEP-based BCI using high-frequency vibration, high-frequency (around 100 Hz) vibration can also induce less tiredness of muscles compared to low-frequency vibration [18, 19]. Accordingly, in the aspects of the interface's usability, the high-frequency SSSEP-BCI can outperform low-frequency regarding long-term usage. Among various types of mechanoreceptors, Meissner's and Pacinian corpuscle receptors are involved in the frequency range of about 100 Hz [20], and the frequency of 100 Hz is suitable for stimulating changes in the human neural system [21]. High-frequency SSSEP-BCI with SA could also help hybridization to decode various EEG intentions [22] due to the frequency range that can be separated from MI (<30 Hz). Thus, high-frequency-based SSSEP BCI could provide more ways of eliciting brain activities to identify various movement intentions.

Various machine learning and pattern recognition-based feature extraction and selection methods have been developed for classifying the SSSEP at a low-frequency range. Nam et al. showed that the band-pass filtering and common spatial pattern- (CSP-) based spatial feature could show higher accuracy than raw signals [23]. Yi et al. suggested a filter-bank CSP- (FBCSP-) based feature extraction method by dividing the raw signal into several frequency bands [24]. Furthermore, FBCSP with the mutual information-based best individual feature (MIBIF) method showed an outperformance for classifying the SA to vibration stimuli attached to the user's left and right hand [14]. The possibility of classifying the user's SA to the high-frequency vibrating stimuli was conducted as a preliminary experiment only using the CSP method [25]; however, there is still a need for more research on applying the high-frequency-induced SSSEP for BCI application [25].

Thus, we aimed to investigate the SSSEP-BCI using vibration stimuli with high frequencies. The main contributions of this study can be summarized as follows. First, we investigated the possibility of classifying the user's SA to vibrating stimuli at high frequencies. In consideration of practical use, vibrating stimuli were implemented with low-cost coin-type motors in our study. In the previous studies, various-type vibration motors (big, heavy, expensive, and sophisticated) were used to elicit SSSEPs at the low-frequency range (<41 Hz) requiring a larger mass [14, 26] but the low-cost coin-type motors can generate the higher-frequency range with a small mass. Second, we compared the decoding accuracy with spatial-spectral feature extraction and selection methods, i.e., CSP, FBCSP, and FBCSP-MIBIF. Our findings can be a basis for further developing the high-frequency vibration-based SA-BCI in real-life appliances.

## 2. Materials and Methods

### 2.1. Experimental Setup

Based on our pilot study during the left and right-hand SA tasks, a sample size of 7 was determined by the power analysis (power = 0.8; *α* = 0.05; effect size *d* = 1.132) using the G∗Power software (ver. 3.1.9.7, Christian-Albrechts-Universität, Kiel, Germany) to detect the effect among the CSP, FBCSP, and FBCSP-MIBIF methods. The power analysis was one of the popular tools to determine the sample size required to detect an effect of a given size with a given degree of confidence [27, 28]. Thus, 7 healthy subjects (age = 28.7 ± 3.5 yrs.) participated in the experiments. All subjects were male and right-handed with no history of neurological disorders. The experiment was approved by the Institutional Review Board at the Korea Institute of Science and Technology, and informed consent was obtained before the experiments from all subjects.

SSSEP signals were acquired via the EEG amplifier (actiCHamp, Brain Products GmbH, Gilching, Germany) with 31 wet-type electrodes (Fp1, Fp2, F7, F3, F4, F8, FC5, FC1, FC2, FC6, T7, C3, Cz, C4, T8, TP9, CP5, CP1, CP2, CP6, TP10, P7, P3, Pz, P4, P8, PO9, O1, Oz, O2, and PO10) according to the international 10/20 system (Figure 1). The ground and reference were mounted at AFz and FCz, respectively. The impedance levels of all electrodes were maintained below 20 k*Ω* during the experiment. Data were acquired at 500 Hz with a lower-pass antialiasing filter at 140 Hz. Then, a 60 Hz notch filter was applied to remove power noise.

The low-cost coin-type eccentric rotating mass (ERM) motor generated sinusoidal vibrotactile stimuli of frequency range from 85 to 127 Hz controlled through the duty cycle of a Pulse Width Modulation (PWM) by the Arduino board (MEGA, Arduino, Somerville, MA) (Figure 1(b)). The vibrating frequencies were measured using an accelerometer (352A71, PCB Piezotronics Inc., Depew, NY) attached to the coin motors.

### 2.2. Protocols for SSSEP Data Acquisition

Before the SSSEP data acquisition, subjects engaged in a screening session to find the resonance-like frequency specified to each subject. This is for finding subject-specific frequency ranges that show the highest power spectrum of EEG signals near the vibration frequencies [29]. We applied vibration stimuli to the subject's left and right index fingers using stimulating frequencies from 85 to 127 Hz in 2 Hz increments for 2 s. The 2 Hz steps were intended consistently, but an error of less than 1 Hz occurred inevitably in each subject. The vibrating frequency was controlled as constantly as possible by the PWM signal, but the difference occurred due to various finger skin compliance in each subject. As a consequence, what we found was that despite the same percentage of the PWM signal, the vibration frequency was different in each subject. Therefore, the vibration frequency was controlled as precisely as possible based on the frequency value obtained from the accelerometer.

In the screening session, based on our previous study [25], specified resonance-like frequencies of each left hand and right hand were found. The resonance-like frequency was the frequency that had the maximum amplitude difference in the EEG signals when the subject gave attention and inattention to vibration [15]. This screening session was implemented for the left and right hands from 85 to 127 Hz in 2 Hz increments. In each screening session for the left or right hand, the subject gave attention or inattention to the vibration motor attached to each index finger of the corresponding hand. For instance, in the screening session for the right hand, with the vibrating motor attached to the right index finger turned on, the subject gave attention or inattention to the vibration motor according to the instructions displayed on the screen (Figure 1(a)), while the vibration motor attached to the left hand was off. When a green circle was displayed on the screen, the subject was instructed to focus their attention on the vibrating motor. When logical reasoning tests or some mathematical problems were displayed, the subject was instructed to focus on solving the tests or problems to avoid paying attention to the powered vibrating motor. In both instructions, the EEG signals were collected and compared to specify the resonance-like frequency for each hand.

After the screening session of each subject, the fast Fourier transform (FFT) was applied to determine each subject-specific resonance-like frequency. The FFT was applied to the acquired EEG data at the C4 channel, and the frequency with the biggest amplitude difference between the attention and inattention task was determined as the resonance-like frequency for the left hand [30]. Likewise, the FFT was applied to EEG data at the C3 channel, and the subject-specific resonance-like frequency for the right hand was determined.

After determining the subject-specific resonance-like frequencies, the subjects selectively attended to one of the vibration stimuli applied on both left and right index fingers by following the commands displayed on the front screen (Figure 1). Each motor provided the vibrotactile stimulation (only one frequency per finger) at each determined resonance-like frequency in the screening session. The left or right arrow was pseudorandomly presented 90 times. A single trial consisted of 10 s (Figure 2(a)), of which a vibratory stimulus was applied for 6 s (Figure 2(b)). Each trial was initiated with a white circle displaying on the screen for 2 s. A green circle was then displayed for 2 s for preparing the SA task. While one of the left or right arrows appeared pseudorandomly for 4 s, the subject performed the SA tasks of the corresponding hand. Finally, a red circle was displayed for 2 s to indicate resting without any stimuli (Figure 2(a)).

### 2.3. Signal Processing and Performance Evaluation

We compared the accuracy of the three feature extraction methods, i.e., CSP [14, 15], FBCSP [14], and FBCSP-MIBIF [14, 31], which showed good performances in the low-frequency SSSEP-BCIs. First of all, the well-known CSP has been specialized for the extraction of spatial features that were distinct between the activating cortices. Therefore, when the left and right-hand SA tasks were performed, the CSP could extract spatial features in the sensory-motor cortex. Furthermore, because the filter-bank strategy could increase the spectral information containing the SA tasks and increase the classification accuracy [14], it was also applied to our study. In the previous studies [31], the FBCSP-MIBIF showed good accuracy in the MI-BCI [31] with reduced computational cost. Therefore, we also investigated the accuracy when the feature selection method was also applied to the high-frequency SSSEP-BCIs.

#### 2.3.1. CSP

The acquired EEG signals were band-passed with 2-120 Hz. The CSP filters were then applied through a one-versus-one (OvO) strategy without any other processing (Figure 3(a)). The logarithmic variances of entire components of the transformation matrix were used as the CSP feature [15, 23].

#### 2.3.2. FBCSP

As shown in Figure 3(b), the acquired raw EEG signals were divided into 7 subfrequency bands; each band size was 10 Hz with 5 Hz overlap (76-85, 81-90, 86-95, 91-100, 96-105, 101-110, and 106-115 Hz). The CSP filters were then applied with the OvO strategy in each subfrequency band. The logarithmic variances of the first and last two components in each CSP transformation matrix (a total of 28) were concatenated and used as the FBCSP feature [14].

#### 2.3.3. FBCSP-MIBIF

The MIBIF algorithm was additionally applied to the FBCSP features (Figure 3(c)). A total of the 28 features were extracted from 7 subfrequency bands. The features were then ranked by the MIBIF algorithm [14, 31]. Consequently, the number of features was selected as 5 pairs referencing the previous low-frequency SSSEP-BCI study [14].

The selected features were finally used for classification using a linear support vector machine (SVM) with a radial basis function kernel algorithm for recognizing the user's intentions (SA to vibrating stimuli on the left or right hand) [3]. Data analyses were conducted using the MATLAB software (MathWorks, Natick, MA).

For performance evaluation, we measured the classification accuracy of 100 bootstrap repetitions with the acquired EEG data composed of an 8 : 2 train-test ratio (Figure 3). The data were randomly sampled with replacement, and the bootstrapped mean was calculated 100 times. In order to obtain a better quantitative comparison between the methods, we performed statistical analysis via the ANOVA with a post hoc test and *t*-test. Bonferroni correction was done for multiple comparisons.

### 2.4. Spectral and Spatial Analysis for the SSSEP

The spectral and spatial characteristics of the SSSEP were also investigated in our study. Each left and right-hand vibration stimuli induce the SSSEP on the contralateral side. According to previous magnetic resonance imaging (MRI) study [32], it is known that the hand's primary motor cortex (M1-Hand) is C3h (positioned between the C3 and C1)/C4h (positioned between the C4 and C2) and C1/C2 within the international 10-5 system [32]. In contrast, the primary somatosensory cortex (S1) of the hand area locates 2 cm posterior and 2 cm lateral to the motor cortex [33]. Therefore, considering the centro-parietal (CP1 and CP2) regions, the bipolar placement (CP1-Cz and Cz-CP2) was used to investigate and visualize the characteristics of the SSSEP more precisely.

## 3. Results

### 3.1. Resonance-Like Frequency

In our study, the screening session was implemented firstly to determine the subject-specific resonance-like frequencies. The determined frequencies for each subject are listed in Table 1. Interestingly, the frequency differences between left and right hand were different for each persons

Figure 4 presents the results of FFT on attention and inattention at the determined resonance-like frequencies of the left and right hand at the corresponding channel (C4: left hand and C3: right hand). There was a significant difference in the amplitude of SSSEP (*p* = 0.0081, effect size = 1.1253) between attention and inattention to vibration stimulation.

### 3.2. Spectral and Spatial Characteristics

In Figure 5, the spectral component of SSSEP was shown from the two opposite areas in the somatosensory cortex. The attention to the left-hand stimuli evoked an increased SSSEP peak (red) on the corresponding vibration frequency (gray peak). The other elevated SSSEP peak amplitude of the right-hand stimuli (blue) was also observed at the same vibration frequency point (black peak). All lines (blue, red, gray, and black) showed the average normalized amplitude from the fast Fourier transform of representative trials within all subjects.

Topological analysis was also conducted to investigate the column factor of the inverse CSP transformation matrix from the difference between the SA to the left and right hand.  Figure 6 shows the representative spatial patterns from all subjects. For the topographies, Figures 6(a) and 6(b) and 6(c) and 6(d) of the CSP transformation matrix at the resonance-like frequencies for each hand were averaged. As a result, when the subjects attended to one of the vibrating stimuli administered to the left hand and the right hand, there were dominant topological differences between the left and right -hand SA tasks.

### 3.3. Classification Performance

We compared the classification accuracy of the CSP, FBCSP, and FBCSP-MIBIF methods with high-frequency SSSEP data.  Figure 7 shows the result of the averaged Bootstrap repetition with a standard deviation. The overall accuracies (binary classification) were calculated as 65.3 ± 1.9% (CSP), 71.5 ± 2.5% (FBCSP), and 67.8 ± 2.3% (FBCSP-MIBIF). Furthermore, ANOVA (*F*(20) = 5.03, *p* = 0.0184) with the Bonferroni post hoc tests revealed that there was a significant difference in the CSP method and the FBCSP method (*t*(12) = −3.096, *p* = 0.0093, and effect size = −1.6546). However, there were no significant differences between the FBCSP method and the FBCSP-MIBIF method and the CSP method and the FBCSP-MIBIF method. According to these results, both the FBCSP method and the FBCSP-MIBIF method outperformed the CSP method.

In the previous study [34], the real level of chance of binary classification in the random classification to BCI was not 50% (theoretical one). When the real level of chance was [34] applied to our study, a random binary classification chance for 40 trials per class in 95% confidence level was 60.1% (statistically estimated, referring to [34]). As shown in Figure 7, the FBCSP method showed a higher performance than the other two methods.

## 4. Discussions

In this study, the feasibility of high-frequency vibrating stimulation for SSSEP-BCI was investigated using low-cost ERM coin-type motors. Distinct spectral and spatial responses of

SSSEP induced by SA to the vibration stimuli were found. The average accuracy of 71.5 ± 2.5% from our study was achieved through FBCSP followed by the SVM classifier. To our knowledge, an average classification accuracy of a tactile SA-BCI experiment with a relatively low-frequency stimulation (19-29 Hz) is also about 69% [26] and 72% [35]. Consequently, our study is valuable because it showed the comparable performance of the previous low-frequency SA studies despite using high-frequency vibration through a low-cost coin-type motor.

As shown in Figure 5, we observed the distinctive spectral component peak of SSSEP measured on the contralateral side of the left and right stimuli in the presence of SA under the high-frequency vibration stimuli. In addition, as shown in Figure 6, the dominant differences in the somatosensory area corresponding to the left and right-hand SA tasks were illustrated by the CSP matrix localizing components in the resonance-like frequencies for each hand. Therefore, in CSP, whereby the EEG signals were band-passed with 2-120 Hz, it is difficult to extract the distinguishable spectral information induced by SA tasks. In FBCSP, the spatial feature (by the CSP) was extracted in each frequency band (76-85, 81-90, 86-95, 91-100, 96-105, 101-110, and 106-115 Hz) and it was concatenated. Thus, due to the characteristics of the spectral and spatial features of our results in the SA tasks, the FBCSP feature extraction method enhanced with a subsequently divided frequency band may show higher classification accuracy than the CSP method (Figure 7).

We expected that employing the MIBIF algorithm could increase the classification accuracy because it showed better performances in a low-frequency SSSEP-BCI study [14]. However, in our study, the MIBIF algorithm did not contribute to improving the classifier's performance. Although the MIBIF algorithm prioritized and selected several specific spectral features (from the divided band-pass filter method; FBCSP) by the amount of information embedded, it may not significantly influence the classifier due to the high-frequency ERM motor characteristic of the widely spanned oscillation range. In a previous study about the MI-BCI, the FBCSP method also showed better performance (79.17 ± 16.73%) in classifying the left and right hand in 9 subjects [36].

Recently, several approaches were investigated for improving the classification accuracy for BCIs [37–39]. Zhou et al. proposed optimizing visual stimulation for increasing the performance of P300-BCIs [39]. With the combination of the tactile stimulation to elicit SSSEP, further research utilizing various visual stimuli could help to optimize stimulation parameters and improve the performance of SA-BCIs. Jin et al. proposed channel selection [37] and feature selection methods [38] for improving the performance of MI-BCIs. Jin et al. proposed the bispectrum-based channel selection method for reducing the effects of noise and redundant information that exists in the multichannel EEG [37] and the L1-Norm and Dempster-Shafer theory-based CSP for improving accuracy. In our study, a channel selection algorithm was not applied while the normal CSP was adapted to extract features. Consequently, the advanced approaches, such as the aforementioned optimizing stimulation parameters, channel selection, and feature selection methods, can be applied to improve the classification accuracy within high-frequency SA-BCI in future work.

Kübler et al. showed that a minimum performance level of 70% is usually required for communication [40]. In our study, the classification accuracy for the high-frequency-based SA showed over the minimum performance level. Therefore, our experimental results of more than 70% classification accuracy are promising. Our approach and results can be a basis for further developing a high-frequency SSSEP-based BCI for controlling external moving devices, such as a wheelchair and lower-limb exoskeleton when utilizing SSVEP-based BCI might be difficult. Furthermore, by adding high-frequency-based SSSEP signals, diverse hybrid BCI classifiers can be developed using diverse frequency features when both MI and high-frequency SSSEP are combined from Mu (8-12 Hz) to the high-gamma band [41, 42].

In future studies, the following supplements are expected to be conducted. First, in order to verify the credibility of our approach, an online experiment can be implemented by controlling a lower-limb exoskeleton via SSSEP-based BCI in real time. The SSSEP induced by high-frequency vibration stimuli should be validated in terms of delay and information transfer rate [43]. Second, the frequency difference between left and right vibration stimuli that induce well-separable SSSEPs should be investigated to reduce the screening session by minimizing the time to find the resonance-like frequency for the effective high-frequency SSSEP-based BCI. Third, to emphasize the usability of the high-frequency SSSEP, the experiments not only with the low-volume coin-type ERM vibrator but also with the widely used mobile devices that embed haptic feedback are warranted. Additionally, adopting a higher sampling rate for the SSSEP acquisition system than the present study is also expected to ensure spectral resolution. Although the number of subjects was determined by our power analysis, seven subjects may not be enough to verify the effectiveness. Therefore, more experiments with a larger population (age, gender, etc.) might be needed for generalizing our findings. At any rate, this is the first study investigating the feasibility of eliciting SSSEP by high vibration frequency for BCI application.

## 5. Conclusions

In this study, considering the real-life appliances, we investigate the possibility of classifying the user's SA as vibrating stimuli with high frequencies using low-cost motors. The experimental results showed that the FBCSP method can classify the high-frequency vibrating stimuli-based SA with higher than 70%. It can be shown that the high-frequency SSSEP could be applied to the BCI protocol for communicating with external devices. In the real-world environment, the performance of each subject can be dependent on various subject-specific factors such as concentration level, and tiredness. Therefore, additional investigation is required to determine how they could affect performance within the high frequency-vibrating stimuli-based SA-BCIs. However, our study is meaningful because it may open up a new door for applying a low-cost SA-BCI paradigm for real-life applications.

## Figures and Tables

**Figure 1:** Experiment environment for (a) steady-state somatosensory-evoked potential (SSSEP) data acquisition and (b) flow diagram illustration. An Arduino board controlled left and right coin motors which were attached to the subjects' index fingers. The accelerometer measured the vibration frequency of the motor. The EEG amplifier transmitted the brain signal and vibration stimuli to the control laptop which managed the experiment procedure.

**Figure 2:** Experiment procedure for left and right-hand SA tasks. (a) illustrates a screen flow that was displayed to the subjects. Each subject randomly engaged in left or right attention of 3 s for 90 trial repetitions (45 trials for each side). (b) shows stimulation of the coin motor which induced vibration frequency to the subjects every 2 to 8 s of the task procedure.

**Figure 3:** An illustration of the SSSEP data processing sequence. The discriminative features were extracted using the FBCSP and were selected using the MIBIF algorithm. Selected features were classified using an SVM classifier. (a) is a shortened process for the CSP data process with a single band-pass and a single spatial filter. (b) is an additional 7 frequency band-pass filter for FBCSP and (c) sequential MIBIF feature selection method.

**Figure 4:** Effect of the attention within the SSSEP amplitude. Each bar indicates the amplitude of attention and inattention to the vibration stimuli at C4: left hand (*L*) and C3: right hand (*R*). The numbers in parentheses also present the resonance-like frequencies of *L* and *R* of each subject.

**Figure 5:** The average normalized amplitude from the fast Fourier transform of representative trials for both EEG signals of CP1-Cz and CP2-Cz electrodes. The red and blue lines depict the SSSEP signals induced by attention to the left and right vibration stimuli on contralateral electrode sites. The left and right accelerometer frequency peaks are illustrated in gray and black bold lines, respectively.

**Figure 6:** Normalized topographies of CSP transformation matrix from all subjects.

**Figure 7:** Bootstrap-based repeated classification accuracy of the CSP, FBCSP, and FBCSP-MIBIF. Each bar with an error bar plot indicates the mean with 1SD from each condition at each person (^∗∗^*p* < 0.01). Values above the gray dotted line (real level of chance of binary classification) considered that the classification accuracy is above the random chance.

**Table 1:** Subject-specific resonance-like frequencies (Hz).

	S1	S2	S3	S4	S5	S6	S7
Left hand	90	94	91	86	88	96	107
Right hand	92	91	87	87	108	91	98

## Data Availability

The original contributions presented in the study are included in the article, and further inquiries can be directed to the corresponding authors.
